# The effect of 3-bromopyruvate on human colorectal cancer cells is dependent on glucose concentration but not hexokinase II expression

**DOI:** 10.1042/BSR20150267

**Published:** 2016-02-19

**Authors:** Nelson Ho, Jodi Morrison, Andreza Silva, Brenda L. Coomber

**Affiliations:** * Department of Biomedical Sciences, Ontario Veterinary College, University of Guelph, Guelph, ON, Canada, N1G 2W1

**Keywords:** 3-bromopyruvate, colorectal cancer, hexokinase II, hypoglycaemia, knockdown, survival signalling

## Abstract

Cancer cells heavily rely on the glycolytic pathway regardless of oxygen tension. Hexokinase II (HKII) catalyses the first irreversible step of glycolysis and is often overexpressed in cancer cells. 3-Bromopyruvate (3BP) has been shown to primarily target HKII, and is a promising anti-cancer compound capable of altering critical metabolic pathways in cancer cells. Abnormal vasculature within tumours leads to heterogeneous microenvironments, including glucose availability, which may affect drug sensitivity. The aim of the present study was to elucidate the mechanisms by which 3BP acts on colorectal cancer (CRC) cells with focus on the HKII/Akt signalling axis. High HKII-expressing cell lines were more sensitive to 3BP than low HKII-expressing cells. 3BP-induced rapid Akt phosphorylation at site Thr-308 and cell death via both apoptotic and necrotic mechanisms. Cells grown under lower glucose concentrations showed greater resistance towards 3BP. Cells with HKII knockdown showed no changes in 3BP sensitivity, suggesting the effects of 3BP are independent of HKII expression. These results emphasize the importance of the tumour microenvironment and glucose availability when considering therapeutic approaches involving metabolic modulation.

## Abstract (precis)

Colorectal cancer cells respond to 3BP via phosphorylation of AKT at residue Thr-308. The availability of glucose in culturing media plays a crucial role in 3BP sensitivity, although independently of HKII expression.

## INTRODUCTION

Tumours up-regulate key glycolytic enzymes to utilize and rely on the glycolytic pathway for energy production regardless of oxygen tension in a phenomenon called the Warburg effect [1,2]. This metabolic strategy promotes tumorigenesis by re-routing glycolytic intermediates to fuel anabolic processes for sustained rapid proliferation [3]. Furthermore, highly glycolytic tumours are associated with disease aggressiveness [4].

The family of hexokinase (HK) enzymes functions to catalyse the first irreversible step of glycolysis in which glucose is phosphorylated to glucose-6-phosphate. Although HK isoforms are differentially expressed in various tissues, HKII is up-regulated in many tumours [5–7]. Mito-HKII promotes metabolic coupling of glycolysis and oxidative phosphorylation while also playing a cytoprotective role by maintaining mitochondrial membrane integrity [8–10].

HKII activity is regulated by the AKT signalling pathway. AKT, or protein kinase B, is a serine/threonine kinase that is often hyperactivated in human cancers. AKT phosphorylates and stimulates the activity of target molecules involved in glucose metabolism, cell proliferation, migration and survival [11–15]. AKT is able to phosphorylate HKII at residue Thr-473 and increase subsequent mitochondrial localization [16,17]. Furthermore, the anti-apoptotic effects of AKT require mitochondrial-bound HKII [18].

3-Bromopyruvate (3BP) is a pyruvate analogue with alkylating properties that depletes cellular ATP levels and induces rapid cell death in neoplastic cells with limited cytotoxic effects against normal cells. 3BP treatment led to eradication of tumours of hepatocellular carcinoma cell origin in rats without apparent cytotoxic effects [19], and the first human case report suggested that 3BP was able to prolong survival in a cancer patient diagnosed with hepatocellular carcinoma in 2012 [19,20]. Other studies have also shown the potential of 3BP as a therapeutic agent in different cancer models, including colorectal [21–23], breast [24], ovarian [25], and pancreatic [26] carcinoma, leukaemia [27], glioblastoma [28,29], malignant mesothelioma [30] and malignant myeloma [31]. 3BP is able to dissociate and inhibit mitochondrial HKII function, thereby reducing ATP production. 3BP binding also frees up binding sites previously occupied by HKII, allowing pro-apoptotic molecules (such as BAX and BAD) to promote the release of cytochrome *c* into the cytosol and induce eventual cell death [27,32]. However, the effects of 3BP on AKT signalling have not been well studied.

In most solid tumours, imbalances between cancer cell proliferation and the angiogenic response lead to some cancer cells being at a great distance from blood vessels. This produces patchy regions of ischemic tumour microenvironment, due to a reduction in both oxygen and nutrient availability, including glucose [33]. Thus, it is important to study not only the impact of oxygen tension on chemotherapeutic resistance, but the effects of hypoglycaemia as well. Xu and colleagues have shown that both HCT116 colorectal cancer (CRC) cells and Raji lymphoma cells grown under hypoxic conditions were more sensitive to 3BP than in normoxia [34], but the effects of glucose exposure on 3BP responses are poorly studied.

In the present study, we examined the effects of 3BP on different human CRC cell lines, with particular emphasis on examining the HKII/AKT signalling axis. We also investigated whether glucose availability plays a role in CRC cell responses to 3BP. We hypothesized that HKII expression would correlate with sensitivity to 3BP exposure in human CRC cells and that a knockdown in its expression would decrease this sensitivity. Furthermore, we hypothesized that decreasing glucose availability would lead to an increase in 3BP resistance due to alterations in metabolic signalling pathways. However, we found that although limiting glucose-media concentrations led to both a reduction in HKII expression and decrease in 3BP sensitivity, direct HKII knockdown via RNA interference did not reduce 3BP sensitivity in CRC cells.

## MATERIALS AND METHODS

### Cell culture and media-glucose reduction

Human CRC cell lines HCT116, CaCo2, SW480 and DLD-1 were obtained from ATCC. Cells were maintained in high glucose (25 mM) Dulbecco's Modified Eagle Medium (DMEM; Sigma–Aldrich) supplemented with 10% fetal bovine serum (FBS; Life Technologies) and incubated at 37°C in a humidified atmosphere containing 5% CO_2_ in room air. Stock 1 M 3BP was prepared in H_2_O, filter-sterilized and aliquots were stored at -80°C for future use.

Cells were routinely maintained under exponential growth by passing them every 3–4 days at a 1/8 dilution. At each passage, media-glucose concentrations were reduced by 2.5 mM, by supplementing no glucose DMEM with 10% FBS and the desired glucose concentration using a sterile stock solution of glucose. Cells were maintained at each reduced media glucose concentration for at least three additional passages before further experimentation.

### Measurement of cell growth

Cell growth assessment was approximated through crystal violet staining. Briefly, 5 × 10^3^ cells were seeded into a 96-well plate and incubated overnight. Cells were then treated with 1–100 μM 3BP for up to 72 h. Post-treatment, media was aspirated and crystal violet solution (1% crystal violet, 20% methanol) was added to each well and incubated for 10 min in room temperature. Plates were then aspirated, rinsed and left to dry overnight. Ten percent acetic acid was used to dissolve the crystals and the absorbance at 590 nm was recorded.

### Protein isolation and western immunoblot analysis

Sodium orthovanadate (1 mM) was added 15 min prior to protein extraction. Following treatment with 3BP or 50 μM etoposide, cells were lysed on ice with lysis buffer (Cell Signaling Technology) freshly supplemented with 2 μg/ml aprotinin, 1 mM phenylmethylsulfonyl fluoride (PMSF) and phosphatase inhibitor cocktail II (Sigma–Aldrich). Samples were centrifuged at 12000 ***g*** for 15 min at 4°C, and supernatant was aliquoted and stored at -80°C for future use. Protein was quantified using the Bio-Rad DC Protein Assay Kit (Hercules, CA). Thirty micrograms of total protein was resolved in a 10% polyacrylamide gel using SDS-PAGE then transferred to a polyvinylidene difluoride (PVDF) membrane. Following transfer, membranes were blocked for 1 h at room temperature in 5% non-fat dry milk diluted in 0.1% Tween 20 in TBS (TBST) followed by an overnight incubation in blocking solution with primary antibodies. After washing, membranes were incubated for 1 h at room temperature with the appropriate peroxidase-conjugated secondary antibody, washed, and subjected to Luminata Forte chemiluminescent substrate (Millipore). Membranes were imaged using the ChemiDoc XRS+ system (Bio-Rad Laboratories) and densitometry was performed using Image Lab software (Bio-Rad Laboratories). Primary antibodies used included rabbit anti-pAkt Ser-473 (9271; 1:1000; Cell Signaling), anti-pAkt Thr-308 (4056; 1:1000; Cell Signaling), anti-pan-Akt (4691; 1:1000; Cell Signaling), anti-caspase 3 (9662S; 1:1000; Cell Signaling), anti-glyceraldehyde-3-phosphate dehydrogenase (anti-GAPDH; AP7873a; 1:1000; Abgent), anti-HKII (2867; 1:5000; Cell Signaling), anti-pPDK1 Ser-241 (3438; 1:1000; Cell Signaling), anti-PDK1 (3062; 1:1000; Cell Signaling), anti-PGK1 (AP7094b; 1:1000; Abgent), anti-PTEN (9188; 1:1000; Cell Signaling), anti-SDH (AP19974b; 1:1000; Abgent), mouse anti-α-tubulin (T5168; 1:200000; Sigma–Aldrich) and rabbit or mouse HRP-labelled secondary antibodies (all 1:20000; Sigma–Aldrich).

### Cell death assay

Cell death was determined through annexin V/PI staining using the Alexa Fluor® 488 annexin V/Dead Cell Apoptosis Kit (Life Technologies) following the manufacturer's protocol. Briefly, 5 × 10^5^ cells were seeded on to six-well plates and incubated overnight. Following 48 h treatment, cells were trypsinized and collected in combination with floating cells. Cell pellets were subsequently washed, resuspended in annexin-binding buffer containing AV and PI dyes and left to incubate for 15 min at room temperature, protected from light. Cells were subsequently analysed using a FACScan™ flow cytometer (BD Biosciences). In total, 1 × 10^4^ events were counted per sample. Fluorescence scatter plots were gated and analysed using the Cyflogic software [35] to determine the percentage of viable and dead cells.

### DNA fragmentation

Following 48 h treatment with 3BP or etoposide, cells were trypsinized, pelleted and stored at -80°C. DNA extractions were carried out using the Omega Bio-Tek Tissue DNA Kit (Norcross, GA) according to the manufacturer's protocol with the following changes: (1) samples were left to precipitate in ethanol overnight, (2) samples were subsequently centrifuged at 6000 ***g*** for 1 min, (3) DNA Wash Buffer step was carried out once and centrifuged for 3 min at 20000 ***g*** for 3 min, (4) samples were eluted in 50 μl elution buffer. DNA samples were run on either a 0.8% or 2% agarose gel at 150 V for 2 h or 100 V for 1.5 h, respectively, and visualized using the ChemiDoc XRS+ system.

### RNA interference

Knockdown experiments were performed by transient transfection of HKII siRNA using INTERFERin (Polyplus-transfections) according to the manufacturer's protocol. Briefly, 5 × 10^4^ cells were seeded into 12-well plates and incubated overnight. Cells were initially transfected with 10 nM siRNA for 24 h in Opti-MEM (Life Technologies) and subsequently allowed to recover in high glucose DMEM for the times indicated. Scrambled siRNA (Sigma–Aldrich) served as a negative control. The sense sequences of double-strand siRNA were previously published [36]:

siHKIIa: 5′-GGAUAAGCUACAAAUCAAA[dT][dT]-3′
siHKIIb: 5′-CGGGAAAGCAACUGUUUGA[dT][dT]-3′

3BP dose response following HKII knockdown was conducted as follows. 2 × 10^5^ cells were seeded into 60 mm^2^ plates and incubated overnight. Cells were transfected with 10 nM siRNA for 24 h in Opti-MEM and subsequently allowed to recover in high glucose DMEM for 24 h. A mixture of both HKII siRNA sense sequences was used. Following cell recovery, a 4 h 3BP dose response was conducted.

### Statistical analysis

Data were presented as means of independent measurements +/− S.E.M. GraphPad Prism v6.0 software (GraphPad Software) was used to perform statistical analysis. One-way ANOVA followed by Tukey's post-hoc tests was performed to determine differences between means within each cell line for flow cytometry and cell growth. Non-parametric Kruskal–Wallis ANOVA followed by Dunn's post-hoc tests was performed to determine differences between means within each cell line for western blot densitometric analysis. At least three biological replicates were used for each analysis unless otherwise specified, and treatments were considered significantly different if a *P* value ≤ 0.05 was achieved.

## RESULTS

### HKII expression is correlated to 3BP sensitivity in human CRC cells

The protein expression of HKII by various human CRC cell lines was evaluated via western blot analysis. All four cell lines showed HKII expression to varying degrees (Figure 1A). HCT116 and CaCo2 cells showed moderate and low HKII expression, respectively, whereas SW480 and DLD-1 cells showed relatively high HKII expression. Corresponding IC_50_ values to 3BP were determined through 72 h crystal violet cell growth assays (Figure 1B) and were as followed: HCT116=22.5 ± 0.7 μM, CaCo2=36.6 ± 2.1 μM, SW480=16.9 ± 1.0 μM, DLD-1=16.9 ± 1.3 μM. 3BP sensitivity of HCT116, SW480 and DLD-1 cells were statistically different from CaCo2, but not from each other (*P*<0.05). Thus, high HKII-expressing SW480 and DLD-1 cells were significantly more sensitive to the effects of 3BP than low HKII-expressing CaCo2 cells.

**Figure 1:** HKII expression is associated with 3BP sensitivity HKII protein expression in CRC HCT116, CaCo2, SW480 and DLD-1 cells was assessed via western blot (**A**). Crystal violet staining assay was used to determine 3BP IC_50_ values in HCT116, CaCo2, SW480 and DLD-1 cells (**B**). IC_50_ values shown represent the means of three biological replicates ± S.E.M.

### 3BP-induced cell death is dose dependent

To determine the cytotoxic effects of 3BP on CRC cells, cell death was measured using AV/PI staining and subsequent flow cytometric analysis. Following 48 h 3BP treatment, cell death was observed in all cell lines examined (Figure 2). Positive labelling with AV was indicative of an apoptotic event whereas PI positivity correlated to a necrotic event. Cells treated with 50 μM etoposide served as a positive control for apoptosis. In all cell lines examined, both forms of cell death were induced upon 3BP exposure. Limited cell death was observed with 5 μM 3BP treatment. At higher doses (30 and 50 μM), the percentage cell death observed in each cell line was associated with levels of HKII expression previously examined. In moderate and low HKII-expressing HCT116 and CaCo2 cells, significant cell death was observed following 50 μM 3BP treatment (56.8 and 26.9%, respectively). In high HKII-expressing SW480 and DLD-1 cells, significant cell death was observed at both 30 μM (31.1 and 78.1%, respectively) and 50 μM 3BP treatment (90.1 and 92.9%, respectively) (Figure 2).

**Figure 2:** 3BP-induced cell death is cell-line dependent Following 48 h 3BP treatment, cell death was assessed through AV/PI labelling and subsequent flow cytometry analysis. Representative plots are shown in (**A**) and quantification of live compared with dead cells from three biological replicates ± S.E.M. are shown in (**B**). Viable cells appear in the lower left quadrant. 3BP-induced significant cell death in all four cell lines (*P≤0.05, **P≤0.01, ***P≤0.001, ****P≤0.0001).

SW480 cells showed considerable caspase-3 cleavage even under control conditions. HCT116 cells were most resistant to etoposide-induced caspase-3 cleavage compared to CaCo2, SW480 and DLD-1 cells. Following 3BP exposure, no cleaved caspase-3 was observed in HCT116 or CaCo2 cells whereas limited caspase-3 cleavage was observed in SW480 and DLD-1 cells (Figure 3A). However, cells exposed to 50 μM 3BP showed overall reduced cellular protein as evidenced by reduced full-length caspase-3 but no detectable cleaved product, and reduced α-tubulin expression. This observation, suggestive of cellular necrosis, was verified using DNA fragmentation analysis, where 50 μM 3BP treatment of SW480 cells led to DNA smearing on the agarose gel, and no obvious nucleosome laddering expected with apoptotic cell death (Figures 3B and 3C).

**Figure 3:** Type of cell death induced by 3BP is dose-dependent Caspase-3 cleavage and DNA fragmentation was assessed to further elucidate the mechanisms of 3BP-induced cell death. Caspase-3 cleavage was examined through western blot analysis (*N*=3) (**A**). An image of a longer exposed membrane to better detect cleaved caspase-3 is shown below each full caspase-3 blot. DNA fragmentation was examined through gel electrophoresis in SW480 cells following 48 h 3BP treatment using 0.8% (**B**) and 2% (**C**) gels (*N*=2). Etoposide (E; 50 μM) was used as a positive control for caspase-3 cleavage and DNA fragmentation; note nucleosome laddering in etoposide treated cells in (**C**) indicative of apoptosis.

### 3BP induces rapid AKT phosphorylation at residue Thr-308

Maximum phosphorylation of AKT at residue Thr-308 was observed after 4 h 3BP treatment (Figure 4A). Dose-dependent changes in AKT phosphorylation following 3BP treatment were observed at residue Thr-308 with no detectable changes at residue Ser-473 (Figures 4B and 4C). Native AKT expression was not affected. The trends in AKT phosphorylation at residue Thr-308 matched the sensitivity to 3BP in different cell lines: phosphorylation occurred at lower doses in cell lines highly expressing HKII (SW480 and DLD-1) (Figure 4C). In CaCo2 cells, AKT phosphorylation appeared to remain constitutively active regardless of 3BP treatment (Figure 4B). Phosphorylation of AKT at residue Thr-308 occurs through PIP3-mediated recruitment of AKT and phosphoinositide-dependent kinase-1 (PDK1) to the plasma membrane [37]. Similar to AKT phosphorylation, changes in PDK1 expression occurred in a dose-dependent manner. Changes in PTEN expression were limited to SW480 and DLD-1 cells, where a decrease in its expression was observed at higher 3BP doses (Figure 4C). At 3BP doses that induced cytotoxic effects, the molecular weight of PDK1 shifted by approximately 3 kDa. In SW480 and DLD-1 cells, an increase in PDK1 expression at higher 3BP doses was observed.

**Figure 4:** 3BP treatment leads to rapid AKT phosphorylation at residue Thr-308 Time course assessment of AKT phosphorylation in response to 3BP. Example from DLD-1 cells shown in (**A**). Western blot analysis of proteins involved in AKT phosphorylation following 4 h 3BP dose–response in HCT116, CaCo2, SW480 and DLD-1 cells (**B** and **C**).

### Glucose availability affects 3BP sensitivity in human CRC cells

HCT116 and DLD-1 cells were adapted to and maintained in DMEM with varying glucose concentrations. Cells were maintained in DMEM containing 25, 5.5 and 1 mM glucose for subsequent experimentation, denoted as ‘high’, ‘normal’ and ‘low’ glucose conditions, respectively. Western blot analysis showed that HKII levels decreased with media glucose levels in both cell lines examined (Figures 5A and 5B). Differences in HKII expression between cells grown under ‘high’ compared with ‘normal’ glucose were more profound in DLD-1 cells. Changes in glucose concentrations did not alter expression of succinate dehydrogenase (SDH), glyceraldehyde-3-phosphate dehydrogenase (GAPDH), nor phosphoglycerate kinase (PGK1) enzymes (Figure 5C). Both CRC cell lines proliferated exponentially under ‘high’ and ‘normal’ glucose concentrations, but growth was limited in cells cultured in ‘low’ glucose over 72 h (Figure 5E). Cells grown in ‘normal’ glucose showed an increase in 3BP resistance compared with cells grown in ‘high’ glucose. Significant differences in cell growth were observed between ‘high’ and ‘normal’ glucose for HCT116 cells treated with 30 and 40 μM 3BP and DLD-1 cells treated with 20 and 30 μM 3BP (Figure 5F). This pattern is consistent with the finding that DLD-1 cells are more sensitive to 3BP than HCT116 cells.

**Figure 5:** Glucose availability alters 3BP sensitivity in CRC cells HCT116 and DLD-1 cells were treated with 3BP under different media glucose concentrations. HKII expression was assessed via western blot analysis. Representative blots from three biological replicates (**A**) and graphical outputs for densitometric analysis of HKII expression normalized to α-tubulin from three biological replicates ± S.E.M. are shown (**B**). Representative blots from three biological replicates of putative 3BP targets SDH, GAPDH and PGK1 show no effects of altered glucose concentrations (**C**). Growth curves for CRC cells grown under different media glucose concentrations in the presence or absence of 3BP over 72 h (**D**). Dose-effects of 3BP on cell growth following 72 h treatment in CRC cells under different media glucose concentrations (**E**) (*P≤0.05, **P≤0.01, ***P≤0.001, ****P≤0.0001 compared with control (0 μM 3BP)).

### HKII knockdown does not lead to changes in 3BP sensitivity

To determine the role of HKII in the differences observed in 3BP sensitivity between different CRC cells, HKII expression was knocked down in HCT116 and DLD-1 cells using transient RNAi transfection (Figure 6A). After 24 h siRNA transfection, media was replaced with DMEM to allow subsequent assessment of 3BP effects in standard treatment media. Protein levels remained knocked down for 48 h post-transfection recovery with a slight increase in HKII expression after 72 h post-transfection recovery (Figure 6B). Given this stability in HKII knockdown for at least 48 h post-transfection, a 4 h 3BP dose–response was conducted on both HCT116 and DLD-1 cells after a 24 h recovery period (i.e. samples were collected for analysis after 28 h knockdown). There were no differences in 3BP sensitivity as revealed by AKT phosphorylation when comparing scrambled siRNA controls to HKII knockdown in either HCT116 (Figure 6C) or DLD-1 cells (Figure 6D). The dose–response patterns observed mimicked those previously seen in parental HCT116 and DLD-1 cells (Figures 4B and 4C), suggesting that, contrary to expectation, a reduction in HKII expression did not lower 3BP sensitivity in the cell lines examined.

**Figure 6:** HKII expression knockdown did not lead to changes in AKT phosphorylation following 3BP exposure HKII expression in HCT116 and DLD-1 cells were knocked down using RNA interference. Both siRNA sequences used showed efficient knockdown of HKII expression following 24 h transfection (**A**). Representative blots from DLD-1 cells are shown. Recovery time of CRC cells following siRNA transfection (**B**). Expression of AKT and related proteins following 4 h 3BP dose–response on HCT116 (**C**) and DLD-1 cells (**D**). siRNA experiments were performed twice with equivalent results.

## DISCUSSION

Although the robust effects of the pyruvate/lactate analogue 3-BP on cancer cells *in vitro* have been well documented, the molecular mechanisms surrounding this remain understudied. We investigated the potential link between HKII expression and the sensitivity of human CRC cells towards 3BP, and whether glucose availability may factor into these cytotoxic effects. Although limiting glucose availability led to a reduction in HKII expression and an increase in 3BP resistance, the expression of HKII alone cannot account for the differences in 3BP sensitivity observed.

Due to its high affinity for glucose compared to other isoforms, HKII is up-regulated during tumorigenesis. This increases glucose consumption and alleviates the metabolic requirements for glycolytic intermediates, thus supporting key anabolic processes that sustain rapid cellular proliferation [5–7]. We examined the expression of HKII in four different CRC cell lines and observed that HKII expression correlated with their reported aggressiveness *in vivo* [38]. Crystal violet was used to monitor effects on cell growth as 3BP has the potential to interfere with the tetrazolium reduction assays (i.e. MTT, WST-1) generally used to evaluate cytotoxicity [39]. AV/PI labelling was used to determine whether 3BP-induced reductions in cell number were primarily due to cell death. In all cell lines treated, a significant portion of cells following >30 μM 3BP exposure appeared in the AV+/PI+ quadrant, signifying either late apoptosis or necrosis [40].

As AV/PI labelling was insufficient to fully elucidate the mechanism of 3BP-induced cell death, we performed additional assays including detection of caspase-3 cleavage and DNA nucleosome fragmentation, both characteristics of apoptotic events [41]. In high HKII expression CRC cells, a slight induction of caspase-3 cleavage following 30 μM 3BP treatment. This effect however was lost with 50 μM 3BP treatment, in which total protein was also reduced, presumably due to microtubule degradation during necrotic cell death. Calvino et al. [42] observed the same trend in myeloid leukaemia cells: increase in cleaved caspase-3 following 30 μM 3BP exposure which was lost at 60 μM. Programmed cell death is not solely dependent on the cleavage and activation of caspases. BH3 domain-only proteins, such as tBID, BIM and BAD can kill cells independently of caspase activation [43]. A common feature in all forms of programmed cell death is DNA fragmentation [41]. However, we were unable to detect the presence of small DNA fragments (representing nucleosomes) in 3BP-treated samples. Instead, there was visible DNA smearing of larger fragments (∼50 kbp) in 50 μM 3BP-treated SW480 cells, suggesting a necrotic event [41]. Combining AV/PI labelling, caspase-3 cleavage, and DNA fragmentation, these results are consistent with apoptosis induction under lower doses of 3BP and necrosis at higher doses.

The specific dose at which 3BP was able to induce these effects was dependent on the cell line. Opinions on the mechanisms of 3BP-induced cell death vary in the literature. Necrosis was induced in both hepatocyte and cancer cell lines following 50 μM 3BP treatment [21,32]. Moreover, a 60% reduction in intracellular ATP levels was observed in hepatoma cells, further suggesting that 3BP induces ATP depletion-dependent necrosis at higher concentrations [32]. In myeloid leukemic cells, both apoptosis and necrosis were induced at 20–30 μM and a pure necrotic response was seen at 60 μM [42], although 3BP is able to induce apoptosis at 100 μM in hepatocellular carcinoma cells [44,45]. The variation observed in 3BP sensitivity and mechanisms of cell death induction may thus be attributed to both the dose and the metabolic phenotype of the cells analysed.

AKT plays a role in the localization of HKII to the mitochondria [17]. In addition to HKII phosphorylation, AKT is able to phosphorylate and inhibit glycogen synthase kinase-3β (GSK3β), a constitutively active serine–threonine kinase able to phosphorylate VDAC and prevent HKII binding. Thus, inhibition of GSK3β leads to increased mitochondrial localization of HKII [46–49]. Initial studies using an approximate IC_50_ dose for DLD-1 showed that Ser-473 of AKT remained constitutively phosphorylated. However, maximum AKT phosphorylation was induced after 4 h of 3BP exposure at residue Thr-308. Rapid induction of AKT phosphorylation following 3BP treatment was previously shown at residue Ser-473 in myeloid leukaemic cells [42]. Changes in AKT phosphorylation at residue Thr-308 correspond with expression of the upstream signalling molecule PDK1. Maximum AKT activity is dependent on phosphorylation of both Thr-308 and Ser-473 residues, the latter of which is phosphorylated by mTORC2 [50,51]. PTEN dephosphorylates PIP3 and prevents AKT membrane recruitment and phosphorylation [52].

Interestingly, we observed a shift in the molecular weight of PDK1 by approximately 3 kDa at cytotoxic 3BP doses. In SW480 and DLD-1 cells, PDK1 expression increased in a dose-dependent manner. Scheid et al. have previously shown that a shift in the molecular weight of PDK1 is a result of hyperphosphorylation in response to survival signalling. Treatment of HEK 293 cells with IGF-1 caused a decrease in PDK1 mobility, and co-treatment with calf alkaline phosphatase reversed this effect, supporting a phosphorylation event [53]. PDK1 is constitutively phosphorylated on at least five serine residues. Residue Ser-241 is located in the activation loops of the PDK1 kinase domain, and its phosphorylation is required for PDK1 activity [54]. Schied et al. [53] also observed that native PDK1 levels reflected the changes in PDK1 phosphorylation at residue Ser-241, and changes in PDK1 phosphorylation reflected changes in AKT phosphorylation at residue Thr-308.

As previously discussed, the *in vitro* conditions used may have a profound effect on the outcome when testing drug efficacy. Since HKII expression is a function of the rate of glucose consumption, we determined whether glucose availability would alter HKII expression and subsequently change 3BP sensitivity. The ‘normal’ glucose concentration (5.5 mM) used for these studies is equivalent to that of normal human physiological steady-state conditions [55], whereas the glucose concentration present in high glucose DMEM (4.5 g/l) is nearly 5-fold greater than what is considered physiological blood sugar levels. We observed a decrease in HKII expression with decreasing glucose concentrations. This change also led to a change in 3BP sensitivity: cells treated in ‘normal’ glucose concentrations were most resistant to the effects of 3BP. It has previously been shown that HCT116 cells induced to exhibit an increased glycolytic phenotype via oligomycin treatment were also more sensitive to the effects of 3BP [22].

Knockdown studies revealed that changes in HKII expression did not lead to altered AKT phosphorylation induced by 3BP. Thus, although high HKII-expressing CRC cells were more sensitive to the effects of 3BP compared with low HKII-expressing cells, this observation cannot explain the differences in 3BP-sensitivity. 3BP affects various enzymes involved in both glycolysis and mitochondrial respiration, including SDH, GAPDH and PGK [56]. It has previously been suggested that an ester derivative of 3BP, 3-bromopyruvate propyl ester, exhibits a more potent inhibitory effect on GAPDH than on HKII in CRC cells HCT116 and HT29 [57]. The ability of 3BP to affect multiple glycolytic enzymes may explain the lack of change in 3BP sensitivity in HKII knockdown cells. However, we saw no alteration in levels of SDH, GAPDH or PGK in our study.

In summary, 3BP is a promising anti-cancer agent capable of inducing rapid ATP loss and cell death in numerous cancer types. We showed that high HKII-expressing CRC cells displayed increased 3BP sensitivity, and that alterations in glucose concentration affected HKII expression and 3BP sensitivity. However, RNAi revealed that HKII expression could not explain the variability in 3BP sensitivity between different cell lines. The mechanism by which lowered glucose concentrations increases 3BP resistance is thus not known. Elucidating the alterations in metabolic pathways that may lead to the observed resistance could provide better understanding of the impact of the tumour microenvironment on CRC cells, and clinical insight to the mechanisms of chemoresistance.

## Abbreviations

3BP: 3-bromopyruvate
CRC: colorectal cancer
GAPDH: glyceraldehyde-3-phosphate dehydrogenase
HKII: hexokinase II
PDK1: phosphoinositide-dependent kinase-1
PGK1: phosphoglycerate kinase 1
SDH: succinate dehydrogenase
